# Computer-Aid Directed Evolution of GPPS and PS Enzymes

**DOI:** 10.1155/2021/6653500

**Published:** 2021-03-18

**Authors:** Fei Chen, Hong Cheng, Jiaqi Zhu, Shiyu Wang, Liancheng Zhang, Haolong Dong, Gang Liu, Huipeng Chen

**Affiliations:** ^1^Institutes of Physical Science and Information Technology, Anhui University, Hefei 230000, China; ^2^School of Life Science and Technology, Dalian University, Dalian 116000, China; ^3^Academy of Military Medical Sciences, Beijing 100850, China

## Abstract

Pinene, a natural active monoterpene, is widely used as a flavoring agent, perfume, medicine, and biofuel. Although genetically engineered microorganisms have successfully produced pinene, to date, the biological yield of pinene is much lower than that of semiterpenes (isoprene) and sesquiterpenes (farnesene). In addition to the low heterologous expression of geranyl pyrophosphate synthase (GPPS) and pinene synthase (PS), cytotoxicity due to accumulation of the monoterpene also limits the production of pinene in microorganisms. In this study, we attempted to use two strategies to increase the biological yield of pinene. By deleting the random coils of GPPS and PS alone or in combination, a strain with a 335% yield increase was obtained. Additionally, upon computer-guided molecular modeling and docking of GPPS with isopentenyl pyrophosphate (IPP), its substrate, the key sites located within the catalytic pocket for substrate binding, was predicted. After screening, a strain harboring the T273R mutation of GPPS was selected among a batch of mutations of the key sites with a 154% increase in pinene yield.

## 1. Background

Pinene (C10H16) is a monoterpenoid compound with a molecular weight of 136.23 Da. According to its features of noncytotoxicity and tastelessness, pinene has been increasingly used in modern industries, such as rubber, coatings, printing, food packaging, and hygiene [1, 2]. There are two isoforms of pinene in nature, *α*-pinene and *β*-pinene, in which *β*-pinene has higher economic value because its double bonds are located outside of the ring to form a dimer more easily [3]. Naturally, existing pinene is mainly produced by the metabolism of coniferous plants, which can secrete turpentine that contains pinene at a percentage of 88% to 95% [4]. Currently, large-scale pinene is acquired mostly from distillation or extraction of turpentine; however, due to the complexity of the turpentine composition, the cost of pinene isolation remains high, but the purity and yield of pinene are relatively low [5].

In the canonical terpenoid metabolism pathway, isopentenyl pyrophosphate (IPP) and dimethylallyl diphosphate (DMAPP), which are essential intermediate products for terpenoid biosynthesis, are transformed to terpenoid precursors catalyzed by isopentenyl transferase, and then, the terpenoid precursors are catalyzed by different terpene synthases (TPSs) to generate various types of terpenoids [6, 7]. Two distinct pathways accounting for DMAPP and IPP synthesis have been identified: the mevalonate (MVA) metabolic pathway and the 1-deoxy-D-xylulose-5-phosphate (DXP) metabolic pathway [8]. Unlike the MVA metabolic pathway, which is ubiquitous in eukaryotic cells [9], the DXP pathway, also known as the methylerythritol phosphate pathway, is limited to some kinds of archaea, animals, most algae, and the chloroplasts of higher plants [10]. For instance, *E. coli* uses the DXP metabolic pathway to synthesize IPP and DMAPP.

To match the increasing industrial demand of pinene, researchers have developed various approaches to improve the yield of pinene at a lower cost and to improve the pinene transformation rate of pinene precursors. In 2013, Yang et al. introduced the MVA pathway into *E*. *coli* combined with extra geranyl pyrophosphate synthase (GPPS) and *α*-pinene synthase (PS) from Abies grandis, followed by a fed-batch culture and fermentation to obtain high *α*-pinene production [11]. In 2014, Sarria et al. linked *Gpps* and *Ps* genes and induced their expression in *E. coli* in a fusion protein mode. The production of pinene increased to 32 mg/L [12]. Moreover, in 2016, by a direct evolution approach, Tashiro et al. obtained an *E. coli* strain harboring manganese-independent GPPS and PS, in which the production of pinene reached 140 mg/L [13]. In addition, some studies demonstrated that GPPS and PS, but not IPP and DMAPP, play key roles in pinene biosynthesis. This is because the levels and activities of GPPS and PS are more essential to the final steps of pinene synthesis than the levels of IPP and DMAPP [14, 15]. Additionally, although overexpression of IPP and DMAPP is easy to achieve, the accumulation of monoterpenes in the cells is usually cytotoxic, and more importantly, excessive plasmids within cells would greatly increase the metabolic burden of the host strains and increase the total number of antibiotic-resistant proteins that have to be introduced, leading to less production of pinene [16]. Notably, the N-terminal sequences within GPPS and PS, which account especially for plastid localization in plants and are then cleaved [17–19], are not indispensable for their catalytic function, indicating that optimizing the length and structure of GPPS and PS in *E. coli* may be a feasible way to improve the yield of pinene in biosynthesis.

Others' and our previous studies revealed that fusion expression of GPPS and PS in *E*. *coli* BL21 is more conducive to pinene synthesis than nonfusion coexpression. Based on that, in this study, we further optimized the activity of the DXP metabolic pathway that was previously established for the *E. coli* strain by using GPPS and PS truncations and point mutations with the guidance of computer informatics to improve the pinene yield. We finally obtained several stains that could produce more pinene.

## 2. Materials and Methods

### 2.1. Prediction of the Secondary Structures of GPPS and PS

The gene numbers for Abies *Gpps* (No. AF513112) and *Ps* (No. U87909.1) were from the Gene Bank (http://www.ncbi.nlm. http://nih.gov/genebank/). The secondary structures of GPPS and PS were generated by PredictProtein online software (http://www.predictprotein.org/).

### 2.2. Molecular Docking of GPPS and the Substrate

The primary three-dimensional (3-D) structure of GPPS was extracted according to homologous alignment in SWISS-MODEL (https://swissmodel.expasy.org/). The stable conformation of GPPS in solvent was obtained by a molecular dynamics simulation and optimization calculation by using NAMD software under the Charmm force field. Then, the 3-D rigid complex structures of GPPS and IPP were acquired by molecular docking using AutoDock software. Considering both hydrophobic interactions and electrostatic effects, among over 30 candidates for GPPS/IPP complex structures, the structure with the minimal energy was selected.

### 2.3. Plasmids

The truncated *Gpps* and *Ps* genes were generated by SOEing PCR, either separately or collectively, followed by linking to the pET-24a vector and transforming *E. coli*. After screening and sequencing, clones harboring correct sequences were selected. Clones encoding wild-type GPPS and truncated PS were named pET24a-GPPS-PStra1 (PS deleted residues 2-38), pET24a-GPPS-PStra2 (PS deleted residues 2-63), and pET24a-GPPS-PStra3 (PS deleted residues 2-80). Clones encoding truncated GPPS and PS collectively were named pET24a-GPPStra-PStra1 (GPPS deleted residues 2-80 and PS deleted 2-38), pET24a-GPPStra-PStra2 (GPPS deleted residues 2-80 and PS deleted 2-63), and pET24a-GPPStra-PStra3 (GPPS deleted residues 2-80 and PS deleted 2-80). GPPS point mutations pET24a-GPPS167R-PS (GPPS167_His-Arg_), pET24a-GPPS138K-PS (GPPS 138_Arg-Lys_), pET24a-GPPS273R-PS (GPPS 273_Thr-Arg_), pET24a-GPPS171F-PS (GPPS 171_Leu-Phe_), and pET24a-GPPS252F-PS (GPPS 252_Ile-Phe_) were generated using a Q5® Site-Directed Mutagenesis Kit (NEB, E0554, MA, USA).

### 2.4. Target Protein Expression in *E. coli*

Engineered *E. coli* strains harboring the GPPS and PS variant vectors described above were cultured in Luria-Bertani (LB) medium with 100 mg/L kanamycin at 200 rpm and 37°C. When the O.D. value of the bacterial medium reached approximately 0.8, IPTG was added at a final concentration of 1 mM, followed by culture for another 10 hours. After that, 0.1 mL of each cell medium was boiled at 100°C for 5 minutes, and then, the supernatant was subjected to SDS-PAGE and Coomassie blue staining.

### 2.5. Determination of the Pinene Yield

The engineered *E*. *coli* strains were cultured using polycarbonate Erlenmeyer flasks (Corning, 430183, NY, USA) and then tested for the pinene content. Briefly, after activation on a small scale, strains were transferred into flasks containing 100 mL of high-density medium with kanamycin and cultured at 200 rpm and 37°C. IPTG was added at a concentration of 1 mM when the O.D. value reached 1.0, and then, the medium was covered with 20% n-dodecane. After culture for another 72 hours at 30°C, the supernatants were harvested to perform pinene detection. The content of *α*-pinene and *β*-pinene in the culture medium was detected by single quadrupole gas chromatography mass spectrometry (Agilent, 5977B GC/MSD, CA, USA) using an Agilent HP-5 MS column. The conditions were as follows: injection port temperature: 200°C; flow rate: 2.5 mL/min, constant flow; split mode: split ratio 50 : 1; column temperature box: start at 50°C, maintain for 3 min, 10°C/min increase to 130°C, hold for 1 min, 130°C/min increase to 280°C, and maintain for 2 min; and injection volume: 1 *μ*L.

## 3. Results

### 3.1. Prediction of the Secondary Structures of GPPS and PS

We obtained the secondary structures of GPPS and PS by using PredictProtein software. As predicted, the random coil of GPPS consisted of N-terminal residues (1-89) (Figures 1(a) and 1(c)). In PS, similarly, residues at the N-terminus (1-85) consisted of a random coil (Figures 1(b) and 1(d)). Although there was a fold sheet structure at residues 48-50, the helix structure was mainly located behind residue 85 (Figures 1(b) and 1(d)). According to previous reports that the random coils of GPPS and PS were unnecessary if not expressed in the plants, we made variants containing GPPS truncation with residues 2-80 lacking and PS truncations with residues 2-38, 2-63, and 2-80 lacking (Figure 1(e)).

### 3.2. Dynamic Analysis and Optimization of GPPS

GPPS and PS are essential to the conversion of terpene precursors to pinene. To achieve our purposes, we modeled the GPPS/IPP interaction complex structure and predicted key sites for the GPPS/IPP interaction. We extracted the GPPS 3-D structure by homologue alignment; however, there were many helix structures in the original modeling conformation of GPPS as well as several atoms positioned improperly within the entire structure. The structure was then optimized in the Charmm force field by taking the protein as the center, adding a spherical water box of 10 *μ*m outside the protein, and adding Na^+^ and Cl^−^ to ensure that the system was electrically eutral. The topology and coordinate structures were preserved during the process. After optimization, loop structures were increased, and the space of groove binding to the substrate was larger (Figure 2(a)). We then modeled the interaction of the optimized GPPS with IPP (Figure 2(b)) by using AutoDock software. During the docking process, over 30 GPPS/IPP complex structure candidates were generated, within which the one with the minimal energy to make IPP stably bind in the groove of GPPS was selected (Figure 2(c)). Three stable hydrogen bonding sites (Figure 2(d)) were identified by kinetic analysis from the binding interface with the substrate. Two strong hydrophobic sites and nine weak hydrophobic sites were identified as well (Table 1). Among them, H167, R138, T273, L171, and I252 were recognized as key sites for IPP interaction. To alter the hydrogen bonding effect, histidine 167 was mutated to arginine, threonine 273 was mutated to arginine, and arginine 138 was mutated to lysine. To alter the hydrophobic interactions, leucine 171 and isoleucine 252 were used instead of phenylalanine.

### 3.3. *E. coli* Expression of GPPS and PS Variants

The catalytic activity of GPPS can be improved by deletion of the random coil. According to the prediction, the “wild-type” GPPS and PS fusion proteins were truncated to different lengths, as indicated in Table 2. Seven truncations were introduced into the BL21 *E. coli* strain, and the strains were named E.G*Δ*80, E.P*Δ*38, E.P*Δ*63, E.P*Δ*80, E.GP*Δ*38, E.GP*Δ*63, and E.GP*Δ*80 (Table 2). In addition, GPPS variants were also obtained and named E.G167R, E.G273R, E.G138K, E.G171F, and E.G252F (Table 2). As visualized by Coomassie blue staining, the variant GPPS and PS fusion proteins were successfully expressed at proper sizes in the corresponding *E*. *coli* strains (Figures 3(a)–3(e)).

### 3.4. Determination of Pinene Yield by GC-MS

The standard curves were made by solutions of *α*-pinene and *β*-pinene with gradient concentrations of 50 ppb, 100 ppb, 500 ppb, 1 ppm, and 10 ppm. The determination of pinene content from various cultured strains was carried out using GC-MS. Compared with the control strain expressing unmodified GPPS and PS fusion proteins, the pinene yield from the engineering strain E.GP*Δ*38 (GPPS*Δ*2-80 and PS*Δ*2-38) was increased to 335% (Figure 4(a)), indicating that deletion of random coils from GPPS and PS significantly improved the pinene production in *E. coli*. Besides that, mutation of threonine 273 to arginine increased the pinene yield up to 154% compared with the control strain (Figure 4(b)).

## 4. Discussion

Terpenes are natural products with high diversity generated by terpene synthase. The distribution of the final products is determined directly by the transformation of carbocation intermediates formed from terpene precursors, which are under the control of terpene synthase. Pinene is produced directly from pinene synthase catalysis of geranyl pyrophosphate (GPP), which is generated from two precursors, DMAPP and IPP, catalyzed by GPPS [6, 7]. Sarria et al. successfully produced pinene in a nonnatural host, *E. coli*, by introducing GPPS and PS. Increased production of pinene in *E. coli* was observed by applying fusion expression of GPPS and PS [12]. However, further improvement of pinene production was confined by the increasing accumulation of GPP in the *E. coli*. Tashiro et al. isolated a mutated pinene synthase from *E. coli* and cyanobacteria by means of directed evolution. Compared with wild-type PS, mutated PS is capable of synthesizing pinene in a manganese ion-independent manner and therefore exhibits better adaptation to diverse chassis cells, indicating enzyme modification as a feasible method [13]. Given that the active pocket of terpene synthase usually shows plasticity to some extent, modification of the residues in the active pocket can change the affinity of the substrate and enzyme and improve enzyme activity [20, 21].

Computer-guided molecular dynamics simulations are widely used to predict key sites responsible for the interaction between two proteins. Under a reasonable force field, the atoms of the interaction interface are dynamically repositioned to form a more reasonable complex structure according to given principles. In this paper, we used this strategy to predict the potential active sites of GPPS bound to IPP to guide further direct evolution of GPPS. We first obtained an optimized GPPS structure with more reasonable atom positioning and a larger substrate binding groove under the Charmm force field. Next, through flexible docking of GPPS and IPP, the complex structures with the lowest phase energy were obtained. As a result, fourteen residues located on the catalyzed groove, potentially bound to IPP, were predicted. Amino acid substitution of these residues could improve pinene production. Among the candidates, after the primary screen, we selected and generated five different GPPS mutations, fused the mutations with PS, and introduced the fusion vectors into *E. coli*. Production analysis showed that T273R exhibited a significant increase in pinene production, while H167R, R138K, L171F, and I252F exhibited moderate increases, confirming the prediction.

In addition, we also constructed fusion proteins consisting of different GPPS truncations and PS truncations lacking N-terminal random coils. N-terminal transport peptides are essential for plastid transportation of translational products in plant hosts; however, they may cause misfolding and disordered localization of the protein itself when heterologously expressed in nonnatural hosts, such as *E. coli*, thus hampering the production of the product [22, 23]. In this paper, we tested pinene production from strains harboring GPPS-PS with GPPS truncation, with PS truncation, or with both truncations. We found that deletion of thirty-eight residues from the N-terminus of PS from GPPS-PS significantly improved pinene production to more than threefold in comparison with the wild type.

## 5. Conclusion

Collectively, we developed a rapid and efficient way to screen “evolutionary enzymes” with higher catalytic activity under the guidance of bioinformatics. By using this method, we obtained two strains harboring modified GPPS and PS fusion proteins that could have higher pinene yields. We provided a new approach to improve the efficiency of pinene biosynthesis, which might contribute to the industrial production of pinene.

## Figures and Tables

**Figure 1:** (a) Protein sequence of GPPS. The truncated part of residues 2-80 is shown in red. (b) Protein sequence of PS. Three parts truncated either alone or combined are shown in purple (2-38), blue (39-63), and green (64-80). (c, d) Predicted secondary structures of GPPS (c) and PS (d). (e) Diagram of variants of the GPPS-PS-truncated fusion protein.

**Figure 2:** Three-dimensional (3-D) modeling of the structure of GPPS and the IPP complex. (a) The optimized 3-D structures of GPPS under a Charmm force field. (b) Schematic depiction of the basic structural features of IPP. (c) Binding of IPP to the substrate binding pocket of GPPS. (d) The predicted key sites in GPPS for IPP interaction. The red and yellow sticks denote the bone structure of IPP, and the green and blue sticks denote key amino acids in GPPS.

**Figure 3:** Expression of GPPS/PS variants in *E. coli*. (a–d) The expression of truncated variants of GPPS/PS fusion proteins in *E. coli*. Lanes labeled with the symbol “+” denote induction by IPTG. (e) The expression of GPPS/PS fusion proteins with GPPS point mutations under induction of IPTG. Ctrl denotes the “wild-type” GPPS/PS fusion protein without IPTG induction.

**Figure 4:** Pinene yields of various engineered strains. (a) Pinene yields of strains expressing GPPS/PS fusion protein truncations. (b) Pinene yields of strains expressing GPPS/PS fusion proteins with point mutations. CK denotes the “wide-type” GPPS/PS fusion protein.

**Table 1:** Key sites for IPP interaction of GPPS and their interaction modes.

Interaction mode	Key site in GPPS
Hydrogen bond in solution	H167
	R138
	T273

Strongly hydrophobic interaction	L171
	I252

Weak hydrophobic interaction	R185
	R186
	I244
	K272
	I268
	K327
	K331
	K337
	D170

**Table 2:** The name and vector information of each strain and what mutation it denotes.

Strain	Vector	Mutation site
E.G*Δ*_80_	pET24a-GPPStra-PS	GPPS*Δ*2-80
E.P*Δ*_38_	pET24a-GPPS-PStra38	PS*Δ*2-38
E.P*Δ*_63_	pET24a-GPPS-PStra63	PS*Δ*2-63
E.P*Δ*_80_	pET24a-GPPS-PStra80	PS*Δ*2-80
E.GP*Δ*_38_	pET24a-GPPStra-PStra38	GPPS*Δ*2-80 PS*Δ*2-38
E.GP*Δ*_63_	pET24a-GPPStra-PStra63	GPPS*Δ*2-80 PS*Δ*2-63
E.GP*Δ*_80_	pET24a-GPPStra-PStra80	GPPS*Δ*2-80 PS*Δ*2-80
E.G167R	pET24a-GPPS_167R_-PS	H167R
E.G273R	pET24a-GPPS_273R_-PS	T273R
E.G138K	pET24a-GPPS_138K_-PS	R138K
E.G171F	pET24a-GPPS_171F_-PS	L171F
E.G252F	pET24a-GPPS_252F_-PS	I252F

## Data Availability

The data used to support the findings of this study are included within the article.

## References

[1] George K. W., Alonso-Gutierrez J., Keasling J. D., Lee T. S. (2015). Isoprenoid drugs, biofuels, and chemicals--artemisinin, farnesene, and beyond. *Advances in Biochemical Engineering/Biotechnology*.

[2] Salehi B., Upadhyay S., Erdogan Orhan I. (2019). Therapeutic potential of *α*- and *β*-Pinene: a miracle gift of nature. *Biomolecules*.

[3] Vespermann K. A., Paulino B. N., Barcelos M. C., Pessôa M. G., Pastore G. M., Molina G. (2017). Biotransformation of *α*- and *β*-pinene into flavor compounds. *Applied Microbiology and Biotechnology*.

[4] Behr A., Johnen L. (2009). Myrcene as a natural base chemical in sustainable chemistry: a critical review. *Chem Sus Chem*.

[5] Chang M. C., Keasling J. D. (2006). Production of isoprenoid pharmaceuticals by engineered microbes. *Nature Chemical Biology*.

[6] Liang P. H., Ko T. P., Wang A. H. (2002). Structure, mechanism and function of prenyltransferases. *European Journal of Biochemistry*.

[7] Keeling C. I., Weisshaar S., Lin R. P., Bohlmann J. (2008). Functional plasticity of paralogous diterpene synthases involved in conifer defense. *Proceedings of the National Academy of Sciences of the United States of America*.

[8] Kuzuyama T. (2002). Mevalonate and nonmevalonate pathways for the biosynthesis of isoprene units. *Bioscience, Biotechnology, and Biochemistry*.

[9] Das A., Yoon S. H., Lee S. H., Kim J. Y., Oh D. K., Kim S. W. (2007). An update on microbial carotenoid production: application of recent metabolic engineering tools. *Applied Microbiology and Biotechnology*.

[10] Kang M. K., Eom J. H., Kim Y., Um Y., Woo H. M. (2014). Biosynthesis of pinene from glucose using metabolically-engineered Corynebacterium glutamicum. *Biotechnology Letters*.

[11] Yang J., Nie Q., Ren M. (2013). Metabolic engineering of Escherichia coli for the biosynthesis of alpha-pinene. *Biotechnology for Biofuels*.

[12] Sarria S., Wong B., Garcia M. H., Keasling J. D., Peralta-Yahya P. (2013). Microbial synthesis of pinene. *ACS Synthetic Biology*.

[13] Tashiro M., Kiyota H., Kawai-Noma S. (2016). Bacterial production of pinene by a laboratory-evolved pinene-synthase. *ACS Synthetic Biology*.

[14] Zhu F., Zhong X., Hu M., Lu L., Deng Z., Liu T. (2014). In vitro reconstitution of mevalonate pathway and targeted engineering of farnesene overproduction inEscherichia coli. *Biotechnology and Bioengineering*.

[15] Dunlop M. J., Dossani Z. Y., Szmidt H. L. (2011). Engineering microbial biofuel tolerance and export using efflux pumps. *Molecular Systems Biology*.

[16] Reiling K. K., Yoshikuni Y., Martin V. J., Newman J., Bohlmann J., Keasling J. D. (2004). Mono and diterpene production in Escherichia coli. *Biotechnology and Bioengineering*.

[17] Turner G., Gershenzon J., Nielson E. E., Froehlich J. E., Croteau R. (1999). Limonene synthase, the enzyme responsible for monoterpene biosynthesis in peppermint, is localized to Leucoplasts of oil gland secretory cells. *Plant Physiology*.

[18] Bohlmann J., Meyer-Gauen G., Croteau R. (1998). Plant terpenoid synthases molecular biology and phylogenetic analysis. *Proceedings of the National Academy of Sciences of the United States of America*.

[19] Köllner T., Schnee C., Gershenzon J., Degenhardt J. (2004). The variability of sesquiterpenes emitted from two Zea mays cultivars is controlled by allelic variation of two terpene synthase genes encoding stereoselective multiple product enzymes. *Plant Cell*.

[20] Morrone D., Xu M., Fulton D. B., Determan M. K., Peters R. J. (2008). Increasing complexity of a diterpene synthase reaction with a single residue switch. *Journal of the American Chemical Society*.

[21] Wilderman P. R., Peters R. J. (2007). A single residue switch converts abietadiene synthase into a pimaradiene specific cyclase. *Journal of the American Chemical Society*.

[22] Burke C., Croteau R. (2002). Geranyl diphosphate synthase from Abies grandis: cDNA isolation, functional expression, and characterization. *Archives of Biochemistry and Biophysics*.

[23] Hyatt D. C., Youn B., Zhao Y. (2007). Structure of limonene synthase, a simple model for terpenoid cyclase catalysis. *Proceedings of the National Academy of Sciences of the United States of America*.

